RETRACTED

# Artificial Intelligence-Based Translation Technology in Translation Teaching

**DOI:** 10.1155/2022/6016752

**Published:** 2022-06-29

**Authors:** Linghui Kong

**Affiliations:** School of Foreign Languages, Lanzhou Jiaotong University, Lanzhou 730070, China

## Abstract

With the advent of the era of artificial intelligence revolution, deep learning is undoubtedly injecting new vitality into machine translation technology. In the context of artificial intelligence, teachers must find new and effective teaching ideas to improve the actual effect of translation teaching, which has drawn the attention of university teachers in recent years. With the development of society and the change of the times, English is becoming one of the implicit requirements of society for talents. Not only in the context of the new changes in curriculum, English teaching in schools and teachers is no longer limited to examinations, but more importantly, it is also significant to cultivate students' comprehensive English ability so that they can really use their English knowledge and solve practical problems in life. On this basis, this paper investigates the practice of teaching English in college in the context of artificial intelligence.

## 1. Introduction

School is an important transition stage for students to learn and grow. In English, students should have the ability to use English flexibly, and teachers should pay more attention to developing students' English speaking and translation skills so as to lay a solid foundation for their future social life and work [1]. Proper use of AI in university English teaching can greatly motivate students, help them to think creatively, and inspire them to actively participate in English learning as translators [2]. Therefore, university teachers are paying more and more attention to it [3]. However, there are still some problems. The lack of special translation courses and specific teaching materials for teaching English in colleges affects the development of students' translation skills. There are some inconsistencies in the teaching process of translation teachers, which are not conducive to the effective improvement of students' translation skills [4].

Secondly, the preparation of university English textbooks focuses on students' basic knowledge and leaves little room for students' thinking, which is mainly manifested in the lack of certain relevance of translation content formulas and the inability to develop targeted translation teaching contents according to students' majors [5]. Although some translation contents are introduced in the arrangement of current university English textbooks, they focus on basic knowledge and lack practical training content for translation skills. In general, the development of students' English translation skills is still missing and needs further research [6, 7].

RETRACTED

Looking back at the history of translation, human translation has been the main method of translation since ancient times. However, with the development of computer technology and the rapid growth of the Internet, machine translation technology is gradually moving into history. As far as the definition is concerned, machine translation (MT) is a technology that can efficiently use computer computing power to convert and transfer information between two languages [8]. The development of machine translation technology has moved from the research stage to the practical application stage. Machine translation is also the main driver of the dynamic development of translation services in the world.

In the field of NLP, deep learning also performs well in tasks such as text summarization, word stem extraction, sentiment analysis, and semantic extraction. Machine translation has a broad application prospect but also possesses certain complexity, so in both academic research and industrial application, machine translation is regarded as a key research task in the field of natural language processing [9–12]. With the advent of the era of the AI revolution, deep learning is undoubtedly injecting new vitality into machine translation technology.

## 2. Related Work

AI technology has now developed to a stage where multiple types of cross-integrated applications are spread across multiple fields, including those related to intelligent scoring technology based on image text recognition and natural language processing. AI has become an effective means of improving efficiency and technology in various industries and will also lead to great changes, and the technology is also affecting the transformation of education and assessment concepts and models in all aspects [13]. The use of AI for scoring is based on social needs. The use of AI scoring is based on social needs, mainly from the development of language testing practices. The current trend of language testing is to improve the authenticity and efficiency of testing, and the introduction of AI technology is essential to improve the authenticity, efficiency, and accuracy of scoring. The main advantages of AI scoring are objectivity, efficiency, and high accuracy. Therefore, in the context of vigorous development of science and technology, national strategies, and the promotion of education informatization, the future of AI will be a major advantage. In the context of developing science and technology, developing national strategies, and advocating informatization of education, it is an inevitable trend that AI technology will be applied to English translation teaching and scoring of writing and translation in the fourth- and sixth-grade exams in the future [14].

RETRACTED

The origin of machine translation can be traced back to the end of the ninth century when Arab cryptologists developed methods of frequency analysis, probability and statistical information, cryptanalysis, and translation into other system languages used in modern machine translation [15]. Although the idea of machine translation originated in the late seventeenth century and the 1920s, [16] proposed a common language in which the same idea is divided into a symbol. In 1956, the first machine translation conference marked a new stage of machine translation research. Since then, scholars around the world began to study machine translation technology. However, there was no significant change in machine translation technology in the following decade.

In 1972, the U.S. Defense Research and Engineering Agency submitted a report showing that their self-developed Logos machine translation system had successfully translated an English military manual into Vietnamese, thus reestablishing the feasibility of machine translation. After this, a succession of researchers made some achievements in machine translation technology [17]. In the late 1980s, the breakthrough of computer hardware quality also brought down the computational cost, the emergence of various machine translation methods marked more significant progress in machine translation, various machine translation competitions began, and machine translation gradually developed from a research topic to practical application [18]. From its origin to the present development, this topic has become hotter and hotter in view of the great research prospect and commercial value of machine translation.

The basic idea is that after inputting the statement to be translated into the EBMT system, the source language statement with the greatest similarity to the input statement is matched in the bilingual corpus instance database, and the corresponding target language translation is generated based on the standard translation of the matched statement. However, the limitation of this approach is that the matching rate is very low and the labor cost is still large [19]. The SMT is to collect a large-scale bilingual parallel corpus, based on which statistics and analysis are performed to construct a useable statistical translation model. The early statistical-based machine translation methods rely almost entirely on word-level modeling with explicit segmentation, which is mainly due to the data sparsity problem, especially for the n-gram networks commonly used in statistical machine translation, where the length of a sequence grows significantly when a sentence is represented as a sequence of characters instead of words, and therefore, statistical machine translation methods are not effective in dealing with long-distance-dependent sentences, or strongly context-dependent passages, and perform poorly [20].

RETRACTED

## 3. Methodology

According to the actual teaching needs, on the basis of AI technology and interdisciplinary foreign language application, the English learning system based on AI consists of four modules: online learning, practical course, intelligent learning management, and intelligent evaluation.

### 3.1. Online Teaching Module

The online teaching module is designed for university English teachers as its main users. In this teaching module, teachers design online courses, display PPT and teaching resources such as audio, video, and microlessons, and provide all texts, vocabulary, explanations, translations, and audio scripts in the form of Word documents, which are informative, interesting, and effective. At the same time, the online teaching teachers focus on sorting out English knowledge for students and consolidating their basic English knowledge. For example, when teaching news listening, teachers will first introduce the structure and style of news, teach students to grasp the general meaning of the news, and also give students a summary of common news topic vocabulary and background knowledge and news listening test-taking skills explanation and analysis; when teaching level 4 reading questions, teachers will carefully explain the six major reading question-solving skills and demonstrate the efficient answer steps one by one, and test preparation experience and test-taking skills will be shared.

### 3.2. Assignment Exercise Module

The homework practice module is for students as its main user. Students can watch high-quality videos, learn texts, memorize words, practice speaking, take tests, and ask questions. This module covers listening, reading, writing, word choice, filling in the blanks, etc. It provides an intelligent review function for essays, and students who study the same course can form a common learning community to compete with each other and learn cooperatively. Through personal homepage and learning dynamic display data, students can show their learning results, share their learning experience, occupy the cover and weekly effort list, so that students can clarify their position and stimulate their learning interest, and also share the learning process by collaborating with each other to complete learning tasks. The exclusive circle of friends based on common learning interests allows students to learn without being alone.

RETRACTED

### 3.3. Intelligent Teaching Management Module

The Smart Teaching Management module also has university English teachers as its main users. This module is able to present all the courses taught by teachers as a list at a glance. Through batch class creation, class announcements, class tasks, learning to monitor, learning statistics, class interaction, batch class closing, and other teaching management functions, teachers are able to track students' learning process in real time, realize online tutoring, test assessment, question and answer discussion for students in this class, and apply big data technology to push important information such as course difficulties and problem students in time.

### 3.4. Intelligent Assessment Module

The intelligent assessment module is a set of intelligent assessment systems covering question bank, machine questioning, and machine marking, which is fully utilized Internet resources and specially designed for non-English majors to take the college English levels 4 and 6 exams. It is a computer-aided foreign language testing system for non-English majors. The graphic recognition technology in the AI can convert students' handwritten compositions and translations into Word documents, which can provide teachers with a large amount of real and effective data for the tutoring and testing of levels 4 and 6. In addition, the objective questions are automatically marked, saving time and efficiency; the subjective questions are manually marked, making the operation convenient.

This module also includes the Panorama English Composition Smart Review Platform. The platform helps English teachers to free themselves from the heavy task of reviewing essays, so that they can focus on teaching English writing test skills and core knowledge, assigning more essay topics for IV exams, allowing students to practice more, and providing targeted tutoring. The machine scoring and intelligent assessment system in this platform not only provides students with a timely and intelligent assessment system but also provides them with objective and accurate composition scores and linguistic, semantic, and grammatical errors in their writing, so that they know the problems and knowledge gaps in their English writing from the very beginning. Over time, they can easily check the gaps, improve their deficiencies, and enhance their English writing; teachers can also get an all-around accurate picture of the overall level of students' English writing in their own classrooms and pay attention to common problems in students' writing. The teacher can also have a comprehensive and accurate understanding of the overall level of English writing of the students in the class, focus on the common problems in students' writing, and then practice a lot with them.

RETRACTED

Taking the English-Chinese translation system as an example, when an original English sentence is input at the input side, the first step is to search all translation alternatives in the pretrained translation model and add them to the cache, and then in the next step, the best translation result is derived according to the language model, and finally the output Chinese translated sentence is obtained through the decoder. The framework structure of the translation system is shown in Figure 1.

In 2014, the sequence-to-sequence (seq2seq) framework was proposed, as shown in Figure 2, in which convolutional neural networks are discarded, both parts of the encoder side and decoder side are composed of RNNs, and long short-term memory networks are introduced to improve the long-distance dependency that may occur during translation, but because the neural networks work on the principle of converting the source language input sequence, the performance cannot be well guaranteed.

The core idea of classical recurrent neural networks is to introduce temporal states, where the hidden state *h*_*t*_ in the current temporal sequence is computed by involving the input *x*_*t*_ of the current temporal sequence and the hidden state *h*_*t*−1_ of the previous sequence, as shown in expression 1. Thus, the hidden state in the current temporal sequence can be used to model the long-range contextual relationships in the text by encoding the sequence content information several temporal sequences ago, a property that fits with the seq2seq framework for machine translation.

(1) $$\begin{array}{c} h_{t}=\tanh\left(W_{xh}x_{t}+W_{hh}h_{t-1}+b_{t}\right). \end{array}$$

In the RNN-based machine translation model, both the encoder side and the decoder side are composed of a single RNN, and the specific RNN machine translation model structure and workflow are shown in Figure 3.

The source language sequence enters the encoder, firstly the word one-hot encoding is transformed by the word embedding layer into the vector space as word vector representation, in this process, the hidden state of each word vector is involved in the calculation of the semantic encoding (context vector *c*) used to record the language information, the semantic encoding is used as the output at the encoder side and the input at the decoder side, and the decoder is involved in the calculation of the hidden state of the decoder. Then, the conditional probability of the target language word is obtained from the hidden state vector, and the word corresponding to the maximum probability is selected from the word list as the word output under the current timing sequence, and the next hidden state is calculated together with the current hidden state and the semantic encoding and the current output as the input. In addition, to facilitate the judgment of whether the language sequence is complete through the neural network model, “<bos>“ and “<eos>“ symbols are added at the beginning and end of the sequence sentences, respectively, to identify the beginning and end of the language sequence.

RETRACTED

The model training process of RNN is actually the process of finding the local maximum of the conditional probability of the output sequence based on the input sequence with the maximum likelihood estimation, as shown in equation (2). In this process, the loss function of the target output sequence is obtained, and the minimization of the loss function is used as the goal for iterative tuning of the network parameters, and expression (3) is the global loss function of the RNN model. Since the recurrent neural network is related to the time series, the parameter iteration is performed using the BPTT algorithm (backpropagation through time), in which gradient descent is used as the optimization method, and expressions (4)–(6) are the parameter gradient update formulas of the recurrent neural network, where *L* is the loss function and *V*, *U*,  and *W* are the three parameters, respectively.

(2) $$\begin{array}{c} \max_{\theta }\frac{1}{N}\sum_{n=1}^{N}\log\;p_{\theta }\left(y_{n}x_{n}\right). \end{array}$$

(3) $$\begin{array}{c} \text{Loss}=\sum_{t=1}^{N}{\mathrm{Loss}}_{t}=-\sum_{t=1}^{N}\left[y_{t}\ln\left(o_{t}\right)+\left(y_{t}-1\right)\ln\left(1-o_{t}\right)\right], \end{array}$$

(4) $$\begin{array}{c} V≔\mathrm{lV}-\eta \frac{\partial L}{\partial V}, \end{array}$$

(5) $$\begin{array}{c} U≔U-\eta \frac{\partial L}{\partial U}, \end{array}$$

(6) $$\begin{array}{c} W≔W-\eta \frac{\partial L}{\partial W}. \end{array}$$

In the decoding stage, the decoder needs to search for the maximum conditional probability of the output based on the input. One method is Exhaustive Search, i.e., the probability of all possible output characters is exhausted, and then the maximum probability of the characters is used to derive the optimal sequence. Exhaustive search can produce the optimal sequence, but it has the problem of excessive computational overhead when the word list is too large. Another common search method is greedy search. Although the greedy search has the advantages of small computational effort and simple computation, it cannot guarantee that the predicted sequence is the most globally optimal. In addition, beam search is also a common search method, whose algorithm idea is to perform width-first traversal in a limited memory space for the search target.

RETRACTED

According to the computational expression of the hidden layer, we know that chain derivation is required during the state propagation of the recurrent neural network. Since the derivative of the ReLU activation function is constant to one in the part of the definition domain greater than zero, the gradient disappearance problem can also be solved by the ReLU activation function.

The attention mechanism-based machine translation model can better focus on the traditional encoder-decoder model that uses fixed-length vectors as sequence encoding vectors. The content restoration and syntactic fluency of the output sequence are improved.  Figure 4 shows the structure of the attention-based machine translation model with a bidirectional recurrent neural network as an example.

The final hidden state *h*_*t*′_ of the encoder is calculated as shown in equation (7), and the resulting context vector *c*_*t*_ is generated as shown in equation (8). *x* is the source language sequence unit input, and *y* is the target language sequence unit output generated by the decoder. The output of each decoder is determined by the state units of all weighted input hidden states and the current timing; *a*_*tt*′_ is defined as the attention weight of how much hidden state information should be considered for each output; e.g., when the value of *a*_32_ weight is relatively large, the decoder pays particular attention to the second hidden state in the source language sequence when generating the third character of the target language sequence. To standardize the representation, the attention weights *a*_*tt*′_ sum up to a value of 1 in the general case, *a*_*tt*′_, and the expression for calculating them is shown in equation (9).

(7) $$\begin{array}{c} h_{t^{\prime }}=\left[{\hat{h}}_{t\prime },{\hat{h}}_{t\prime }\right], \end{array}$$

(8) $$\begin{array}{c} c_{t}=\Sigma_{t^{\prime }=1}^{T}a_{tt^{\prime }}h_{t^{\prime }}. \end{array}$$

(9) $$\begin{array}{c} a_{tt{\;}^{\prime }}=\frac{\exp\left(e_{tt{}^{\prime }}\right)}{\sum_{t\prime =1}^{Tx}\exp\left(e_{tt{}^{\prime }}=\alpha \left(s_{t-1},h_{t{}^{\prime }}\right)\right)}, \end{array}$$

where *e*_*tt*′_ is defined as the attention score calculated for each hidden node at the output of the encoder to indicate the degree of influence of the characters in the encoder at *t*′ timing on the characters in the decoder at *t* timing, as shown in equation (9), where *α* can be defined as a variety of alignment models, such as dot product matrix and multistring mapping.

RETRACTED

The transformer is the dominant framework in neural machine translation and is the first sequence-to-sequence model to compute its input and output representations using only a self-attentive mechanism, also using an encoder-decoder architecture. The basic idea is to use the recursive computation of the attention mechanism to handle the dependencies between the source and target sequences. Since RNNs are discarded and data features cannot be abstracted dynamically in terms of temporal sequences, relative position information is added to this framework. Its encoder and decoder ends are actually multiple identical encoders and decoders stacked on top of each other, with a single decoder/encoder containing only the self-attention layer and feedforward layer, and a multiheaded attention layer in both the encoder and decoder ends. The advantage of using multiheaded attention is that it enables the model to focus on information from different locations. Therefore, the number of encoders and decoders is one of the hyperparameters. A diagram of its framework structure is given in Figure 5.

The word embedding of the input sequence to the first encoder is first passed to the first encoder and then propagated to the next encoder through the self-attentive layer and the feedforward network, thus forming an iterative network. The attention layer creates a query vector (*Q*), a key vector (*K*), and a value vector (*V*) based on the word vector of each input to the encoder, from which the attention weights of all words in a sequence are calculated with respect to the current word. The output of the attention layer is calculated as shown in expression (10). The multiheaded attention layer is used to project query vectors, key vectors, and value vectors using multiple linear transformations, and then, the results are integrated.

(10) $$\begin{array}{c} {\text{attention}}_{\text{output}}=\text{soft}\max\left(\frac{QK^{T}}{\sqrt{d_{K}}}\right)V. \end{array}$$

The last encoder in the encoder stacking end passes its output state vector to all decoders in the decoder stacking end as contextual encoding input, so the decoder end outputs the probability distribution of characters at corresponding positions with the output vector of the encoder and the upstream output of the encoder as input. In the decoder, in addition to the self-attention layer and the feedforward layer, there is a multiheaded attention layer in the decoder, which serves to ensure that the current predicted values in the training phase are not disturbed by other information so that the decoder focuses on the appropriate segments of the input sequence.

(11) $$\begin{array}{c} e_{tt{}^{\prime }}=\alpha \left(s_{t-1},h_{t{}^{\prime }}\right). \end{array}$$

RETRACTED

## 4. Experiment

The experiments in this section aim to implement and compare the current mainstream deep neural network machine translation models, and due to the practical situation, this experiment uses a small-scale English-Chinese bilingual parallel corpus dataset as the experimental data; the translation task language direction selects the English to Chinese direction; the development framework selects the deep learning framework TensorFlow; the development experiment model selects several basic neural network translation models, which are recurrent neural network model, long short-term memory network model, and bidirectional recurrent neural network model, and adds attention mechanism to the above models, where transformer uses Tensor2tensor as its implementation framework. Other parameters are set to the same size, and the details are described in the following section.

The experimental dataset is compiled from the public dataset (wmt-18-news-commentary) and the Internet provided by the International Conference on Machine Translation (WMT2018) in the category of news commentary. Since the purpose of the experiments in this chapter is to compare the advantages and disadvantages of several networks and to select the optimal model to adjust the parameters, the dataset is set small. It is divided into a set of 500,000 English-Chinese parallel sentence pairs as the training set, a set of 2,000 English-Chinese parallel sentence pairs as the validation set, and two sets of 1,000 English-Chinese parallel sentence pairs as the test set. The datasets are organized as shown in Table 1.

Based on the principle of comparing different network models, the hardware and software environment and other experimental parameters are set as constant conditions except for the network model which is set as variable conditions. The development environment is shown in Table 2 and some parameters are shown in Table 3.

With the same development environment and parameter settings, the mainstream statistical machine translation model Maverick statistical machine translation model is selected as the baseline system to compare with the neural network model as a comparison; RNN, LSTM, and bidirectional recurrent neural network model (BiRNN) are constructed for training according to the above parameters, and the attention mechanism algorithm, together with the transformer model, is used for comparison. The results of this experiment are given in Table 4.

The table shows the BLEU-4 scores of this experiment, which illustrates the effectiveness of machine translation models based on deep learning neural networks, and the performance of several networks in machine translation tasks based on comparative experiments. From the results obtained in the validation set and the two test sets, firstly, several neural network-based translation models have BLEU scores that exceed the baseline system, among which transformer has the highest BLEU-4 score; among the models that do not incorporate the attention mechanism, the long short-term memory network translation model has the best performance, followed by the bidirectional recurrent neural network model, and finally the unidirectional recurrent neural network model. From the control group of the four networks incorporating the attention mechanism, the performance of each translation model after incorporating the attention mechanism showed considerable improvement, and the inclusion of the attention mechanism significantly reduced the gap with the baseline.

RETRACTED

From the above, we can conclude that the transformer model is the best performing model. In order to provide a reference for the next experimental parameters for the data size of this paper, a parameter comparison experiment was designed based on the transformer model. The experimental design is as follows: the word table size is modified to 16000 and 32000, respectively, and the two models are retrained based on the transformer framework using the dataset in Table 1 and tested on the two test sets for comparison. The experimental results are shown in Table 5.

The contents of the above table show that the model with a word list size of 16000 has an average improvement of 2.3 points on BLEU-4 over the model with a word list size of 8000, while when the word list size is 32000, it has a decrease of 1.67 points over the word list size of 8000. Represented by a line graph as in Figure 6, the line graph allows us to see more intuitively the effect of word table size setting on the model performance.

The following analysis can be derived from the results of this experiment: the word list size has a certain influence on the performance of the neural machine translation model, but it does not grow linearly with the word list size, and after the word list size exceeds a certain size, it reduces the model performance instead. The reason for this analysis may be due to the limitations of the BPE algorithm of the rare word processing method itself. For example, when the word table is set too large, some illegal characters will be added to the word table, which will affect the translation performance. Therefore, it can be concluded that appropriately adjusting the word table size within a certain range according to the size of the dataset can help improve the model performance.

RETRACTED

In Figure 7, we show the changes in students' satisfaction with English translation teaching courses before and after the application of artificial intelligence technology. It can be seen that students' satisfaction has been improved to varying degrees before and after application. Further, we show the preference of different modes of teaching practice in the hearts of students in Figure 8. It can be seen that the teaching method of AI is more popular.

## 5. Conclusion

In the context of AI, the practice of English translation teaching in colleges and universities needs to be changed, and teachers in colleges and universities need to adopt scientific and effective strategies through in-depth reflections and comprehensive discussions to effectively integrate AI with English translation teaching practice in colleges and universities, so as to cultivate all-round talents, contribute to the development of society, and promote the future development of translation science in a positive direction. If a high-quality translation environment can be created with the help of AI technology, it is to create favorable conditions for our university students to improve their English translation skills. This will ensure greater achievements in English subject education in our higher education institutions, thus ensuring that students can achieve all-round development and improve their overall quality while mastering translation skills.

## Figures and Tables

**Figure 1:** Framework of the statistical machine translation system.

**Figure 2:** Framework of seq2seq model.

**Figure 3:** RNN machine translation model structure.

**Figure 4:** Diagram of the structure of the attention mechanism machine translation model.

**Figure 5:** Schematic diagram of the structure of the attention mechanism machine translation model.

**Figure 6:** BLEU-4 folding line diagram.

**Figure 7:** The satisfaction of different students.

**Figure 8:** The comparison of different teaching modes.

**Table 1:** Experimental dataset settings.

Dataset settings	Scale/thousand lines	Quantity/group
Training set	500	1
Validation set	2	1
Test set	1	2

**Table 2:** Development environment settings.

Development environment	Name
GPU	GeForce GTX TITAN
Development system	UBUNTU
Development language	Python3. 7
Deep learning framework	TensorFlow, tensor2tensor

**Table 3:** Parameter settings.

Parameter type	Parameter
Word list size	8000
Word vector dimension	515
Batch size	1024
Number of network layers	6
Dropout	0.2
Learning rate	0.1
Optimizer	Adam
Beam search width	5

**Table 4:** Translation model BLEU-4 score table.

Model	Validation set	Test set 1	Test set 2
Calf translation	11.33	11.00	10.76
RNN	11.95	11.22	10.89
LSTM	13.57	12.71	12.58
BiRNN	12.36	12.24	12.04
RNN + Attention	15.45	15.15	14.57
LSTM + Attention	16.30	15.83	15.68
BiRNN + Attention	15.61	15.44	15.53
Transformer	18.37	17.91	17.19

RETRACTED

**Table 5:** Word table size comparison experiment BLEU-4 score table.

Thesaurus size	Validation set	Test set 1	Test set 2
8000	18.35	17.89	17.17
16000	20.51	20.07	19.29
32000	16.57	16.21	15.55

## Data Availability

The experimental data used to support the findings of this study are available from the corresponding author upon request.
